The article "Meta-Analysis for Social Support Degree of Kidney Transplant Recipients: Evidence from China" was retracted in 2023. Reasons: unreliable results or conclusions; concerns about the data; concerns about the peer review; concerns about the citations.

# Meta-Analysis for Social Support Degree of Kidney Transplant Recipients: Evidence from China

**DOI:** 10.1155/2021/9998947

**Published:** 2021-08-12

**Authors:** Qiaolan Yang, Min Xia, Shaohua Hu, Yazheng Chen, Guiyi Liao

**Affiliations:** ^1^Institute of Urology, The First Affiliated Hospital of Anhui Medical University, Anhui Medical University, Hefei 230022, Anhui, China; ^2^Nursing Department of the First Affiliated Hospital of Anhui Medical University, Anhui Medical University, Hefei 230022, Anhui, China; ^3^Department of Gynecology and Obstetrics, West China Second University Hospital, Sichuan University, Chengdu 610041, Sichuan, China

## Abstract

Social support refers to the subjective and (or) objective influence of various social relationships on individuals, which has a certain influence on the negative emotions of the kidney transplant patients. But there are still significant differences among various studies, so we performed a meta-analysis to analyze the social support degree of kidney transplant recipients. This article searched and selected the relevant cross-sectional surveys from PubMed, Embase, VIP, CNKI, Wanfang, and CBM databases according to the inclusion and exclusion criteria and used the STROBE list combined with the observational research quality evaluation tools of Sanderson to conduct the quality appraisal. The “meta” and “metaphor” packages of the R software version 3.5.1 were used for the meta-analysis. A total of 17 studies with 2697 patients were included. The total scores of the social support and objective support of the renal transplant patients were abundant after the operation, indicating that the economic, physical, and emotional supports from the family, society, and the official organization are accepted. But the subjective support and support utilization degree were general. The support utilization was different among different genders, and female patients were lower than the males. In particular, the female patients relatively presented autism and the social support utilization degree was low. Medical staffs are needed to join the family, hospital, and society to create favorable conditions and improve the social support system and the utilization degree of the social support, thereby promoting the physical and mental health development of the patients.

## 1. Introduction

Kidney transplantation is the radical and most effective conventional treatment for the end-stage renal disease (ESRD) [1]. Globally, in 2017, there were 697.5 million cases of Chronic Kidney Disease (CKD) [2]. With 132.3 million CKD patients, China is the country with the biggest number of patients in the world [2]. At present, the number of transplantations in China ranks second in the world, next only to the United States [3]. Kidney transplant recipients may experience various negative emotions due to the long-term treatment and the particularity of recovery process after transplantation. The rejection reactions and various complications after the operation with the long-term treatment and the expensive costs bring about heavy psychological pressure as well as disease uncertainty to the kidney transplant recipients. These negative emotions may significantly affect recipients' psychological health and quality of life. Effective social support can relieve these negative emotions.

The article "Meta-Analysis for Social Support Degree of Kidney Transplant Recipients: Evidence from China" was retracted in 2023. Reasons: unreliable results or conclusions; concerns about the data; concerns about the peer review; concerns about the citations.

The concept of social support was first proposed in the field of psychiatry. Social support received wide attention in the 1970s–1980s and later became a generic term in many disciplines [4]. Objective support refers to visible or actual support, including material assistance and the participation of social groups. Subjective support refers to the emotional experience and satisfaction of an individual being respected, supported, and understood in society, which is closely related to the one's subjective feelings [5]. Utilization of social support refers to the degree to which the individuals utilize the social support. Some individuals may have access to social support but refuse it [5]. Social support is reciprocal in nature. When one gives support to others, he or she is more likely to receive support from others as well. The social support rating scale (SSRS), developed by Xiao et al. in 1986, consists of three dimensions: objective support (3 items), subjective support (4 items), and support-seeking behavior (3 items). The higher the total score and the scores of each dimension, the higher the level of social support [6].

Significant differences existed among various studies conducted on social support for kidney transplant recipients. There is still a lack of meta-analysis of social support among these patients. In the present study, we reviewed the existing studies on the social support for kidney transplant recipients. A meta-analysis was performed for domestic and foreign studies on the social support for kidney transplant recipients. Our aim was to reveal the facts about each dimension of the social support for these patients. We believe that our findings will shed light on improving psychological status and quality of life in kidney transplant recipients from the perspective of social support.

## 2. Materials and Methods

### 2.1. Literature Retrieval and Search Strategy

The following Chinese databases were searched: VIP Chinese Citation Database, China Knowledge Resource Integrated Database (CNKI), Wanfang Database, and China Biology Medicine disc (CBM). The search was conducted using terms related to kidney transplantation and social support. The terms related to social support were support, social support, level of social support, and social support rate scale (SSRS). These terms were combined by OR and then connected with “kidney transplantation” by AND. The foreign-language databases searched included the PubMed and Embase databases. The search words were “social support” OR “support” OR “social support rate scale” OR “SSRS” AND “kidney transplantation” OR “renal transplantation” OR “kidney transplant” OR “renal transplant.” The time range searched was from inception to November 2019.

The article "Meta-Analysis for Social Support Degree of Kidney Transplant Recipients: Evidence from China" was retracted in 2023. Reasons: unreliable results or conclusions; concerns about the data; concerns about the peer review; concerns about the citations.

### 2.2. Inclusion and Exclusion Criteria

Inclusion criteria: (1) studies were on social support among kidney transplant recipients at home and abroad; (2) SSRS was used for social support assessment; (3) cross-sectional study design was adopted; (4) studies included subjects who had undergone a kidney transplant since three months or more; (5) studies were published in Chinese or English.

Exclusion criteria: (1) literature reviews, conference papers, case reports, and dissertations; (2) included subjects who had severe diseases and complications, such as disability, paralysis, organ dysfunction, underlying complex chronic diseases, mood disorders, mental illnesses, and senile dementia; (3) studies that did not offer complete data on the level of social support among the kidney transplant recipients.

### 2.3. Literature Screening Workflow

First is the preliminary screening: the titles and abstracts of the studies were reviewed, and those that obviously did not satisfy the inclusion criteria were eliminated. Second is the rescreening: the full texts of the studies passing the preliminary screening and the studies with ambivalent screening results were reviewed. Third is the quality assessment: the preliminarily included studies were subject to quality assessment, and the low-quality studies were excluded. Fourth is the literature screening, which was done by two researchers independently, with cross-checks. Any divergence of opinions was settled through discussion.

### 2.4. Data Extraction

Data were extracted by two researchers independently after reading the full texts. A database was built using Excel, and the following information of the studies was sorted and extracted: title, first author, year of publication, survey area, sampling method, sample size, survey tool, average age, percentage of male and female subjects, and outcome indicators. The data extracted by the two researchers were cross-checked. Any inconsistency was settled by discussion or by judgment from the third party.

The article "Meta-Analysis for Social Support Degree of Kidney Transplant Recipients: Evidence from China" was retracted in 2023. Reasons: unreliable results or conclusions; concerns about the data; concerns about the peer review; concerns about the citations.

### 2.5. Outcome Indicators

The variables finally included in the meta-analysis included the SSRS total score, objective support, subjective support, and utilization of social support. The norms were determined according to the report by Cheng et al. [7].

### 2.6. Quality Assessment of the Included Studies

Quality assessment was done by combining the methods section of STROBE Checklist V4 Cross-Sectional with the quality assessment tools for observational studies by Sanderson et al. Ten dimensions (12 items) were used to assess the study quality: study design, setting, participants, variables, data sources, bias, sample size, quantitative variables, statistical methods, and conflict of interest. Each item was assessed as either mentioned (Y) or not mentioned (N).

### 2.7. Statistical Analysis

SMD and its 95% confidence intervals (CIs) were estimated for the pooling of studies. Heterogeneity across the included studies was assessed using the *I*^2^ index and Cochran's *Q* test. A value of *I*^2^ > 50% or *P* < 0.05 indicated significant heterogeneity across the studies. The random-effects model was used if there was heterogeneity; otherwise, the fixed-effects model was used. Metaregression analysis was conducted to explore the sources of heterogeneity. Egger's test and Begg's test were used to detect publication bias. Sensitivity analysis was performed by excluding one study at a time. All analyses were carried out using the “meta” and “metaphor” packages of the R software version 3.5.1. *P* < 0.05 was considered as a significant difference.

## 3. Results

### 3.1. Basic Features of the Included Studies

Figure 1 shows the process of literature search and screening. A total of 204 studies were identified through database search, and 84 studies were identified after deleting duplicates. After quality assessment, 17 studies were finally included for meta-analysis.

Table 1 shows the main characteristics of the included literature. 15 of the 17 studies described the SSRS total score, objective support, subjective support, and utilization of social support, and 2 of them only reported the SSRS total score. These studies were published from 2002 to 2019, and a total of 2697 patients were included, including 1758 males and 939 females, aged 40.39 ± 4.82 years.

### 3.2. Results of the Meta-Analysis

Figure 2 shows the heterogeneity test result of the 17 research literatures on the SSRS total score, suggesting that there is significant heterogeneity among these studies (*I*^2^ = 91%, *P* < 0.01). A random-effects model was used to assess the data and we found that the SSRS level was significantly increased in patients after renal transplantation (SMD = 0.35; 95% CI = 0.20–0.50; *P* < 0.05). There is significant heterogeneity among the 15 research literatures with objective support, subjective support, and utilization of social support (*I*^2^ = 85%, *P* < 0.01; *I*^2^ = 92%, *P* < 0.01; *I*^2^ = 85%, *P* < 0.01, respectively). Compared with the norm, the random-effects model was used and we found that objective support (SMD = 0.57; 95% CI = 0.44–0.70; *P* < 0.05) and subjective support (SMD = 0.19; 95% CI = 0.01–0.36; *P* < 0.05) significantly increased, but no difference was found in utilization of social support (SMD = 0.06; 95% CI = −0.06–0.19; *P* > 0.05). The details are shown in Figures 3–5.

The article "Meta-Analysis for Social Support Degree of Kidney Transplant Recipients: Evidence from China" was retracted in 2023. Reasons: unreliable results or conclusions; concerns about the data; concerns about the peer review; concerns about the citations.

Metaregression analysis was used to explore the possible causes of heterogeneity.  Table 2 shows the results of the metaregression analysis, suggesting that the number of females in patients may be the source of the heterogeneity in the SSRS total score among the studies (*P*=0.026), and the remaining features were not found to be possible causes of heterogeneity (*P* > 0.05).

### 3.3. Sensitivity Analysis

Figure 6 shows the results of the model sensitivity analysis. After removing each study in turn, the total analysis results of the model had no significant changes, indicating that the meta-analysis results were more robust.

### 3.4. Publication Bias

Table 3 shows that Egger's test and Begg's test of the SSRS total score, objective support, subjective support, and utilization of social support showed no significant publication bias (*P* > 0.05).

## 4. Discussion

Family and social supports for the patients undergoing kidney transplants have become a growing concern among medical staffs due to the recent development in family medicine and continuous nursing. Kidney transplant recipients can get material support and also emotional support from society. Social support plays a vital role in alleviating anxiety, depression, and disease-related stress. Social support is closely related to human health. Earlier studies showed that a higher level of social support was beneficial for health [25–28]. On the contrary, a lack of social support was harmful to the health. Quality of life (QOL) is an important indicator to evaluate the therapeutic effect and mortality of kidney recipients. Studies have shown that, compared with the general population, the QOL of kidney recipients was worse [29], and the availability of social support was an independent risk factor for QOL of kidney recipients, indicating that the higher the availability of support, the higher the QOL [30]. Our meta-analysis of multiple studies indicated significant differences in the postoperative SSRS total score and the objective support in the kidney transplant patients compared to the norms (*P* < 0.05). To be more specific, the kidney transplant patients had full access to material assistance, social network, and group relations. Previous studies have demonstrated that gender, age, educational level, social status, work, living conditions, marital status, and learning are important influencing factors of social support available for kidney transplant patients [8–11, 13, 14].

The article "Meta-Analysis for Social Support Degree of Kidney Transplant Recipients: Evidence from China" was retracted in 2023. Reasons: unreliable results or conclusions; concerns about the data; concerns about the peer review; concerns about the citations.

Subjective support refers to how individuals perceive, accept, or feel towards care and assistance from the outside world. The greater the individuals' perceived support is, the stronger the confidence to fight the disease will be, and hence the individuals can be more likely to adopt a health-promoting behavior. On the contrary, the lower the level of perceived support is, the more likely the patients will suffer from such negative mentality as pessimism and self-abasement. As a result, the patients are more susceptible to low subjective well-being and poor quality of life [5]. Kidney recipients need to take antirejection medicine for the rest of their lives, in addition to regular follow-up, and suffer from high sociopsychological stress related to transplantation at the same time, such as the high medical costs, the burden of self-monitoring and management, and the change of lifestyle and social role [11]. The level of their anxiety and depression is obviously higher than that of normal people [30]. Pisanti et al. [31] had shown that social support had a moderating effect on the relationship between high transplant-related stressors and anxiety and had a buffering role on the patients' distress following kidney transplantation, which suggested that their psychological well-being could benefit from enhancing the perception of social support in postoperative care. Tao et al. [32] showed that the patients' utilization of social support was enhanced by a more profound development and mining of the social support system. In such cases, the patients can better integrate into society, forgetting about their diseases and finally becoming healthy kidney recipients. Our meta-analysis found no significant differences in the subjective support and utilization of social support in the kidney transplant recipients compared to the norms (*P* > 0.05). In other words, the kidney transplant recipients had a low level of subjective support. Moreover, they did not fully accept or utilize the social support available to them, including the economic, material, and emotional assistance from family, social groups, and official organizations. Medical staffs should provide appropriate intervention in the clinical practice to enhance the subjective support and utilization of social support among the patients with kidney transplantation.

The article "Meta-Analysis for Social Support Degree of Kidney Transplant Recipients: Evidence from China" was retracted in 2023. Reasons: unreliable results or conclusions; concerns about the data; concerns about the peer review; concerns about the citations.

The suddenness, uncertainty, and continuity of the public health emergency often cause people to suffer from great psychological pressure, and they are even troubled by panic, anxiety, depression, restlessness, irritability, and other emotions [33]. Deng et al. [34] showed that anxiety and depression of the public increased during the COVID-19 pandemic, among which 34.3% and 44.2% of the public showed moderate-to-severe level of anxiety and depression. Transplant recipients may selectively adhere to different tasks depending on the value and priority they attach to potential side effects and complications [35]. During the COVID-19 pandemic, restrictions on the traffic and outpatient services at public hospitals exhibited an adverse impact on the follow-up visits, treatment, and psychology of patients. Family and social supports are crucial for the rehabilitation of the patients undergoing a kidney transplant since such supports provide psychological relief and channel negative emotions in these patients. At present, the risk of COVID-19 still exists worldwide, and further researches are recommended.

The assessment of methodological quality as part of a systematic review is widely recommended but is also still a matter of ongoing debate. Most principles of a systematic review are the same for both randomized controlled trials and observation designs [36]. However, there is no validated or widely used criteria list for observational studies available, so we composed a checklist specifically for this review. We computed a method score for internal validity and reporting separately to overcome the problem that positive scores on descriptive criteria compensate for shortcomings in internal validity. Still, within the list for internal validity, the disadvantage of equal weight for each criterion may lead to the high ranking of studies despite major flaws in methodology [37–39].

Therefore, the nursing staffs should improve the cognition of social support, try to include patients' social support system in health education so as to provide a better support system for them, and work closely with families, hospitals, and other social resources to create favorable conditions for these patients. Support, care, and assistance need to be provided to the patients through multiple pathways. Besides, more efforts should be made to improve the existing social support system. Additionally, patients receiving kidney transplant should be fully informed of the importance of social support for their physical and psychological health and spend more time with their relatives and friends. These measures could enhance the level of subjective support and the utilization of social support for patients with kidney transplantation.

The article "Meta-Analysis for Social Support Degree of Kidney Transplant Recipients: Evidence from China" was retracted in 2023. Reasons: unreliable results or conclusions; concerns about the data; concerns about the peer review; concerns about the citations.

This meta-analysis still has some limitations. First, in the literature search, only Chinese and English documents that have been publicly published were searched. We did not include unpublished and gray documents. Second, with few literatures in the end and lack of high-quality papers, there is no subgroup analysis of different sources of donated organ, which may influence the results. Finally, we mainly analyzed the social support status of kidney transplant patients but did not summarize measures to improve subjective support and the utilization of social support analysis, because there were no systematic solutions in the original papers. Further studies can extend to multicenter patients to help find out the influence factors of social support. Besides, researches can develop optimum comprehensive plans related to improving social support and explore the application effects in the future.

Taken together, our conclusions are based on the meta-analysis by integrating identified studies, which were more reasonable in guiding the medical practice. However, because SSRS is developed by Chinese researchers and is not fully corroborated by foreign studies, more relevant studies are needed to guide the medical practice better.

## Figures and Tables

**Figure 1:** Meta-analysis workflow.

**Figure 2:** Forest plot of the SSRS total score.

**Figure 3:** Forest plot of the objective support.

**Figure 4:** Forest plot of the subjective support.

**Figure 5:** Forest plot of the utilization of social support.

**Figure 6:** Sensitivity analysis diagram.

**Table 1:** Characteristics of samples.

No.	Author	Year of publication	Regions	Samples	Age	Male/female	SSRS total score (mean, standard deviation)		Objective support (mean, standard deviation)		Subjective support (mean, standard deviation)		Utilization of social support (mean, standard deviation)	
1	Zeng [8]	2019	Fujian	226	39.99	150/76	40.33	6.35	9.80	4.01	24.36	5.06	6.07	2.10
2	Sun et al. [9]	2018	Anhui	170	38.00	141/29	41.74	5.10	10.13	1.48	23.28	4.24	7.42	1.62
3	Wu [10]	2018	Shandong	314	38.61	218/96	43.24	8.43	10.71	3.77	25.14	5.14	7.39	2.13
4	Liu and Jiang [11]	2017	Sichuan	252	32.36	198/54	43.43	7.68	10.48	3.35	25.03	4.72	7.92	1.86
5	Wang [12]	2016	Xinjiang	100	41.58	75/25	40.67	8.41	12.76	4.41	24.22	6.59	6.69	2.02
6	Li et al. [13]	2014	Shaanxi	164	51.95	121/43	44.15	8.04	11.15	3.28	25.88	4.84	7.12	1.99
7	Yang and Liu [14]	2011	Guangzhou	145	45.00	88/57	42.31	9.65	10.21	2.95	24.90	7.23	7.33	1.76
8	Lei et al. [15]	2010	Hunan	123	37.60	84/39	42.89	8.48	10.27	3.88	25.28	5.34	7.35	2.05
9	Lei [16]	2010	Hunan	162	39.30	114/48	44.20	8.07	11.11	3.46	25.98	4.91	7.11	1.95
10	Zhang et al. [17]	2009	Guangzhou	203	39.86	130/73	38.34	1.80	9.94	2.52	21.19	4.67	7.20	1.80
11	Zhou et al. [18]	2009	Shaanxi	60	35.00	37/23	43.21	5.63	9.58	2.67	25.76	5.11	7.95	1.89
12	Liu et al. [19]	2008	Sichuan	37	35.00	8/29	36.10	7.80	10.39	3.80	17.38	4.97	8.33	2.01
13	Liu et al. [20]	2007	Beijing	446	47.60	247/199	38.34	2.25	-	-	-	-	-	-
14	Liu [21]	2006	Beijing	141	44.55	65/76	41.28	7.62	10.26	3.01	23.60	4.54	7.42	2.41
15	Luo [22]	2005	Beijing and others	60	41.00	40/20	38.67	8.87	8.92	3.75	22.25	5.74	7.50	2.15
16	He and Guan [23]	2004	Sichuan	58	40.90	30/28	44.18	5.88	-	-	-	-	-	-
17	Cai et al. [24]	2002	Zhejiang	36	38.39	12/24	40.08	8.47	11.81	4.19	21.19	6.14	7.16	2.14

The article "Meta-Analysis for Social Support Degree of Kidney Transplant Recipients: Evidence from China" was retracted in 2023. Reasons: unreliable results or conclusions; concerns about the data; concerns about the peer review; concerns about the citations.

**Table 2:** Results of the metaregression analysis.

Variables	SSRS total score		Objective support		Subjective support		Utilization of social support	
	Coefficient (95% CI)	*P*value	Coefficient (95% CI)	*P*value	Coefficient (95% CI)	*P*value	Coefficient (95% CI)	*P*value
Year of publication	−0.018 (−0.069–0.032)	0.069	0.014 (−0.046–0.073)	0.6525	−0.001 (−0.772–0.074)	0.9713	−0.030 (−0.072–0.012)	0.166
Number of males	0.005 (−0.001–0.011)	0.075	−0.0002 (−0.007–0.006)	0.956	0.005 (−0.003–0.013)	0.216	0.002 (−0.003–0.007)	0.399
Number of females	−0.009 (−0.017–−0.001) 0.018	0.026	−0.003 (−0.014–0.007) 0.015	0.567	−0.006 (−0.020–0.008) 0.030	0.411	−0.004 (−0.011–0.004) −0.019	0.370
Age	(−0.015–0.052)	0.278	(−0.022–0.052)	0.427	(−0.017–0.077)	0.216	(−0.045–0.007)	0.151

**Table 3:** Egger's test and Begg's test.

Dimensions	*t*-value	*P* value	*Z* value	*P* value
SSRS total score	0.184	0.857	−0.330	0.742
Objective support	0.404	0.693	0.049	0.961
Subjective support	−1.803	0.095	−1.732	0.083
Utilization of social support	0.803	0.437	0.544	0.586

## Data Availability

The data supporting this meta-analysis are from previously reported studies and datasets, which have been cited. The processed data are available from PubMed, EMBASE database, VIP Chinese Citation Database, China Knowledge Resource Integrated Database (CNKI), Wanfang Database, and China Biology Medicine disc (CBM).
